# Class A **β**-Lactamases as Versatile Scaffolds to Create Hybrid Enzymes: Applications from Basic Research to Medicine

**DOI:** 10.1155/2013/827621

**Published:** 2013-08-28

**Authors:** Céline Huynen, Patrice Filée, André Matagne, Moreno Galleni, Mireille Dumoulin

**Affiliations:** ^1^Laboratory of Enzymology and Protein Folding, Centre for Protein Engineering, Institute of Chemistry, University of Liege, (Sart-Tilman) 4000 Liege, Belgium; ^2^ProGenosis, Boulevard du Rectorat, 27b-B22, (Sart-Tilman) 4000 Liege, Belgium; ^3^Laboratory of Biological Macromolecules, Centre for Protein Engineering, Institute of Chemistry, University of Liege, (Sart-Tilman) 4000 Liege, Belgium

## Abstract

Designing hybrid proteins is a major aspect of protein engineering and covers a very wide range of applications from basic research to medical applications. This review focuses on the use of class A **β**-lactamases as versatile scaffolds to design hybrid enzymes (referred to as **β**-lactamase hybrid proteins, BHPs) in which an exogenous peptide, protein or fragment thereof is inserted at various permissive positions. We discuss how BHPs can be specifically designed to create bifunctional proteins, to produce and to characterize proteins that are otherwise difficult to express, to determine the epitope of specific antibodies, to generate antibodies against nonimmunogenic epitopes, and to better understand the structure/function relationship of proteins.

## 1. Introduction

Engineering proteins with improved properties or new functions is an important goal in biotechnology. In this context, numerous bi- or multifunctional proteins have been created for applications in a broad range of fields including biochemical analysis, protein purification, immunodetection, protein therapies, vaccine development, functional genomics, analysis of protein trafficking and analysis of protein interaction network [1]. The most common strategy to create such proteins involves fusing polypeptides into an end-to-end configuration. For example, the fusion of proteins with specific tagging domains is nowadays a standard tool for protein engineering. Indeed, numerous commercial kits allow the fusion of a protein of interest to an affinity polypeptide such as 6-Histidine tag, maltose-binding protein, and glutathione transferase [1]. Moreover, the fusion of a protein of interest to the green fluorescent protein (GFP) has become one of the most important tools used in contemporary bioscience, and O. Shimomura, M. Chalfie, and R. Y. Tsien were rewarded the Chemistry Nobel prize in 2008 for the initial discovery of GFP and development of important GFP-based applications.

Another strategy to create hybrid proteins, although much less commonly used, is to insert (or graft) a peptide/protein/fragment thereof at a permissive site of a carrier protein. For example, Collinet et al. [2] have successfully created bi- or trifunctional hybrid enzymes by inserting the dihydrofolate reductase (159 aa) and/or the TEM-1 *β*-lactamase (263 aa) into four different positions of phosphoglycerate kinase (415 aa). Betton et al. [3] have created hybrid proteins by inserting the TEM-1 *β*-lactamase at various sites into the MalE maltodextrin-binding protein, that is, positions 120, 133, and 303, or by fusing it to the carboxy terminus of MalE. Insertion at positions 133 and 303 or fusion at the C-terminus allows the production in the periplasm of hybrid proteins exhibiting both parental activities; indeed, the maltose binding and the penicillinase activity of these hybrid proteins is indistinguishable from that of, respectively, MalE and TEM-1 [3]. Interestingly, the two proteins with insertions displayed two additional properties compared to their C-terminal fusion counterpart: (i) they were more resistant to degradation by endogenous proteases and, (ii) even more remarkably, the TEM-1 moiety was stabilized against urea denaturation through the binding to MalE of maltose, that is, its natural ligand. This latter observation clearly demonstrates that TEM-1 is structurally dependent on MalE or in other words that an allosteric interaction occurs between the two proteins [1, 3]. Thus, insertion of a polypeptide inside a scaffold protein can present some advantages compared to the more common end-to-end fusion. This strategy actually mimics that used by nature to generate protein diversity. Indeed, genetic rearrangements, such as the introduction of a sequence into an unrelated coding sequence, naturally occur in the genome [2]. The resulting proteins are composed of two or more domains, and the linear sequence of one domain is interrupted by the insertion, forming discontinuous domains. This process has been shown for large natural proteins such as disulfide bond isomerase A (dsbA) [4], DNA polymerase [5], and pyruvate kinase [6]. A systematic survey of structural domains showed that ~28% of them are actually not continuous, clearly indicating that the sequence continuity of a domain is not required for correct folding and function [2, 7].

In this review, we report the use of two class A *β*-lactamases to create hybrid proteins (*β*-lactamase hybrid proteins, BHPs) in which exogenous peptides/proteins/fragments thereof are inserted within *β*-lactamase sequences. Such hybrid proteins can be designed for a range of applications such as (i) the creation of bifunctional hybrid proteins [8–11], (ii) the production, purification, and characterization of proteins otherwise difficult to express [10, 12, 13], (iii) the determination of the epitope of a specific antibody at the surface of an antigen [8, 11], (iv) the generation of antibodies against specific antigens or fragments thereof [9, 13–15], and (v) the investigation of fundamental aspects of structure, stability, and function of proteins [10, 12, 16].

## 2. Class A **β**-Lactamases as Scaffolds to Create Hybrid Enzymes

### 2.1. Why the Use of Class A *β*-Lactamases?

The two class A *β*-lactamases that have been extensively used as model proteins to insert exogenous polypeptides are BlaP from *Bacillus licheniformis* 749/C and TEM-1, the latter being the most encountered *β*-lactamase in gram-negative bacteria (Figure 1). These two enzymes are, respectively, secreted by bacteria in the external environment and expressed in the periplasmic space to inactivate *β*-lactam antibiotics. About 40% and 20% of the amino acids are, respectively, identical and homologous between these two serine-active *β*-lactamases (Figure 1). Note that the residue numbering used in this review is that specific to class A *β*-lactamases [17]. These enzymes, especially TEM-1, have been extensively used as reporters to study gene expression [21–23] and for immunoassays [24]. They have been selected as scaffolds to create hybrid proteins based on a series of observations. Firstly, they are fairly small (30 kDa) and stable proteins that are easily overexpressed in *E. coli* and subsequently purified [9–11]. Their three-dimensional structure has been determined by X-ray crystallography (Figure 1) [18, 19, 25, 26]. They exhibit the typical class A *β*-lactamase 3D structure which is composed of two domains: an *α*/*β* domain and an all-*α* domain, with the catalytic site at the interface between the two domains [19, 25, 26]. Finally, their catalytic properties have been thoroughly characterized and can be easily monitored using fluorescent [22, 23, 27] or chromogenic substrates [28]. This latter point is crucial as exemplified in the following sections. The enzymatic activity of the BHPs serves as a reporter to select clones resistant to *β*-lactam antibiotics, such as ampicillin, expressing well-folded and active BHP. It is assumed that the folding of the exogenous polypeptide and the carrier enzyme are interdependent to some degree. Indeed, the correct folding of the carrier *β*-lactamase requires the exogenous polypeptide to be exposed to the solvent; otherwise, the *β*-lactamase cannot adopt its native structure. Moreover, the correct folding of the carrier protein imposes constraints at the N- and C-terminal extremities of the inserted polypeptide, maintaining its two extremities in close proximity of the insertion site. These constraints limit therefore the conformational flexibility of the insert and could assist the insert in adopting its native structure. When a greater flexibility is required for the correct folding of the insert, small peptides, that is, linkers, can be added at both of its extremities. Note that, in some applications, these linkers have an additional functionality allowing the excision of the insert thereafter, as discussed in detail below.

### 2.2. A Brief History of Class A *β*-Lactamase Hybrid Proteins

The design of class A hybrid *β*-lactamases was initiated with the work of Hallet et al., in 1997 [20]. A random pentapeptide cassette was inserted at 23 different positions of TEM-1 using pentapeptide-scanning mutagenesis (Figure 1(a)) [20]. This method consists of transposing the transposon Tn*4430* into the TEM-1 gene which duplicates 5 base pairs (bp) of host sequence at the insertion point. This transposon contains *Kpn*I restriction enzyme sites 5 bp from the outer ends of its terminal inverted repeats. Digestion with *Kpn*I followed by ligation results therefore in the insertion of 10 pb derived from Tn*4430* and 5 bp from the 5-nucleotide duplication of the target gene. Each transposition event leads to a 15 bp insertion into the TEM-1 gene encoding for a random pentapeptide cassette. The 23 insertion sites have been classified into 3 groups depending on the level of resistance that the hybrid protein confers to *E. coli* cells against ampicillin, a *β*-lactam antibiotic (Figure 1(a)): (i) 5 permissive sites (197, 198, 265, 270, and 272) with high level of resistance. These sites are located into two loops distant from the catalytic site, one loop between *α* helices 8 and 9 and the other between *β*-strand 5 and the C-terminal helix. (ii) Eight non-permissive sites (63, 68, 163, 164, 208, 232, 233 and 246) associated with the loss of the *β*-lactamase activity and clustered around the catalytic site. (iii) Ten semi-permissive sites (37, 97, 99, 119, 206, 216, 218, 260, 264, and 276) are conferring an intermediate level of ampicillin resistance. 

Later, Ruth et al. [9] have inserted longer and more structured polypeptides in eight of the TEM-1 positions investigated by pentapeptide-scanning mutagenesis (Table 1). The thermostable 18-residues STa enterotoxin from enterotoxic *Escherichia coli* has been introduced, for example, into one of the two permissive loops (at position 195 and 198, between *α* helices 8 and 9), in five semi-permissive sites (37, 206, 216, 218 and 260) and into one non-permissive site (232). Insertions between *α* helices 8 and 9 (positions 195–200) and between *α* helices 9 and 10 (positions 213–220) allow the production of a soluble hybrid protein which retains both activities of parental proteins (i.e., ampicillin resistance and enterotoxicity). The level of activities and the amount of soluble hybrid enzymes produced depend however on the position of insertion.

TEM-1 is a *β*-lactamase sensitive to many proteases [11, 29]. Some BHPs that do not confer resistance to ampicillin to *E. coli* (i.e., BHPs containing insertions at sites identified as non-permissive) could however be successfully expressed in protease-deficient *E. coli* strains. This observation suggests that insertions at these positions into TEM-1 actually increase its sensitivity to proteolysis [11]. This increased susceptibility to proteolysis could be due to local conformational changes or to a destabilisation of the enzyme upon the insertion of the exogenous polypeptide. In contrast, BlaP presents an advantage over TEM-1 in being much less sensitive to proteases. Indeed, this enzyme evolved to withstand high levels of various and numerous proteases, which are secreted by the gram-positive *Bacillus licheniformis* bacterium [11, 30]. Based on this observation, it was anticipated that BlaP could constitute an alternative scaffold to TEM-1 to generate hybrid proteins. Since, as mentioned above, BlaP and TEM-1 share a high sequence identity and a similar three-dimensional structure, the permissive sites described for TEM-1 served as a basis to engineer hybrid BlaP proteins with the insertion of heterologous polypeptides (Figure 1(b)) [11]. 

### 2.3. How Were BHPs Designed?

TEM-1 hybrid proteins were produced in the periplasm of *E. coli* via pFHX plasmids derived from the pBR332 plasmid, the X corresponding to the position of insertion into TEM-1. These plasmids carry a *KpnI* restriction site at the position of insertion allowing the insertion of the exogenous sequence. They allow a constitutive expression of the BHPs which are purified by ion-exchange chromatography [9].

Most BlaP hybrid proteins, on the other hand, have so far been created by inserting the exogenous polypeptide at position 197 within the permissive loop located between the *α* helices 8 and 9 (Figure 1(b)) [10]. A constitutive expression vector in *E. coli* (pNYBlaP), which allows the insertion of heterologous polypeptide sequences into the *SmaI *restriction site at position 197 (Figure 1(b)), has been developed [10, 11]. This vector allows the expression, in the periplasm of *E. coli*, of the BHP in fusion with a C-terminal His-tag to facilitate their purification using affinity chromatography. 

## 3. BHPs as Tools to Produce and Study Difficult to Express Peptides/Proteins

Some proteins are difficult to produce recombinantly because of their intrinsic properties such as relative insolubility, instability and/or large size. One strategy to study their properties (i.e., structure, function,…) consists of inserting these proteins or their structural subdomains into a carrier protein.

Vandevenne et al. [10] have, for example, designed, produced, and characterized a hybrid protein in which the chitin binding domain (ChBD) of the human macrophage chitotriosidase has been inserted in BlaP at position 197; this hybrid protein is referred to as BlaP-ChBD (Table 1). The study of the chitin binding domain of this chitinase is of interest since (i) the physiological function of mammalian chitinases remains unknown [31] and, more importantly, (ii) the concentration of chitotriosidase, a chitinase expressed in lipid-laden macrophages, is highly elevated in Gaucher disease [31–33]. Some evidence suggests that mammalian chitinases confer a defensive function against chitin-containing pathogens, such as fungals, which have cell walls consisting mainly of chitin; indeed, high levels of chitinases are present in the serum and tissues of guinea pigs after infection by *Aspergillus fumigates *[31, 34, 35]. It is also proposed that the enzyme could modulate the extracellular matrix in the vessel wall affecting the downstream tissue-remodelling processes, associated with atherogenesis. This hypothesis is based on the fact that macrophages expressing chitinases are abundant in atherosclerotic plaques [31, 33].

ChBD is a small domain of 8 kDa composed of 72 amino acids which binds insoluble chitin. It contains 3 disulfide bridges that are essential for both its structural stability and its binding to chitin [10, 13, 31]. This protein domain is extremely difficult to produce, and its three-dimensional structure has not yet been solved [10, 13, 31]. 

The BlaP-ChBD hybrid protein has been successfully produced in the periplasm of *E. coli *and purified in a two-step procedure, that is, affinity chromatography via a His-tag designed at the C-terminus of BlaP, followed by anion-exchange chromatography. Remarkably, the hybrid protein exhibits both parental activities (Table 1). The *β*-lactamase moiety hydrolyzes its *β*-lactam substrates, in the presence and/or absence of chitin, and the ChBD domain binds to insoluble chitin with similar *K*_*r*_ value (relative equilibrium association constant), 5.4 ± 0.5 L g^−1^, of other carbohydrate-binding domains [10, 13]. It is important to note that the bifunctionality of the hybrid protein allowed the *K*_*r*_ value between BlaP-ChBD and insoluble chitin to be easily measured, using the *β*-lactamase activity as a reporter. Moreover, the hybrid protein allowed the detection of chitin in fungal cell walls [24]. The fact that ChBD conserves its binding properties within BlaP suggests that its N- and C-terminal extremities are proximal in the three-dimensional structure. In the presence of reducing agents, BlaP-ChBD still exhibited *β*-lactamase activity but failed to bind to chitin, confirming that the 3 disulfide bridges of ChDB are essential to maintain its functionality. 

The effects of the insertion of ChBD on the thermodynamic stability of BlaP were extensively characterized. Despite the multidomain character of BlaP-ChBD, urea unfolding occurs according to a simple two-state mechanism and is fully reversible [10]. The insertion of ChBD in position 197, however, slightly destabilizes BlaP by 3.2 kJ·mol^−1^ (Table 1). Moreover, the thermal unfolding of BlaP-ChBD was found to be less reversible and less cooperative than that of BlaP. Indeed, the thermal transition observed for BlaP-ChBD by differential scanning calorimetry (DSC) and far UV circular dichroism is characteristic of a three-state transition while the one observed for BlaP is characteristic of a two-state transition. This suggests that, within the hybrid protein, ChBD and BlaP unfold individually upon temperature increase [10]. 

The ChBD domain has also been inserted in position 197 of BlaP between two thrombin (Thb) cleavage sites; this hybrid protein is referred to as BlaP-*Thb/CHBD/Thb* (Table 1) [13]. This construction allowed easy separation of the ChBD domain from the BlaP carrier protein, following the action of the thrombin and subsequent purification. Upon proteolytic cleavage, the N- and C-terminal parts of BlaP remain strongly linked together and are separated from the ChBD domain by depletion using affinity chromatography via the C-terminal His-tag (Figure 2). Remarkably, the thrombin cleavage did not significantly alter either the activity of BlaP or that of of ChBD (Table 1), and ~18 mg of highly soluble and active ChBD was obtained per litre of culture [13, 24]. 

These studies clearly demonstrate that BlaP is an efficient scaffold to create bifunctional enzyme and to produce, purify, and characterize protein fragments that are otherwise difficult to express. This approach has been further used to produce various polypeptides of up to 40 kDa in size (unpublished results). Moreover, these results show that the BHPs can be used (i) to easily investigate the biological function of the polypeptide/protein inserted such as its interaction with a series of ligands using the *β*-lactamase activity as a reporter, (ii) to screen therapeutic molecules, that is, molecules neutralizing the biological properties of the polypeptide inserted, as further exemplified in the section of this review describing the use of BlaP for vaccine development, (iii) to screen molecules stabilizing and preventing protein aggregation (see section “BHPs as model proteins to investigate structure/function relationships”), and (iv) to facilitate the determination of the three-dimensional structure of polypeptides that are otherwise unnameable to X-ray crystallography due to their insolubility, since BHPs allow an increase in the solubility of the insert [10, 12, 13]. 

## 4. BHPs: An Original Approach to Map and Functionalize Epitopes

The determination of the epitope (i.e., the region of the antigen that is recognized by an antibody or an antibody fragment, which can be linear or conformational) is of crucial importance to understand, at the molecular level, the relationship between the structure and function at the antigen-antibody interface [8]. For example, the determination of the epitope recognized by two heavy-chain antibody fragments specific to human lysozyme has allowed a better understanding of how they prevent *in vitro* amyloid fibril formation by the amyloidogenic variants of human lysozyme [36, 37]. Moreover, the identification of the epitope enables the design and isolation of new antibody analogues, having higher affinity for their antigen or exhibiting different biological activities, or smaller antibody mimetics (i.e., peptides and small molecules interacting with the same epitope region) [8]. Epitope mapping is also essential in diagnostic, immunotherapy, and vaccine development. 

Different techniques have been developed to identify epitopes. The gold standard for epitope identification is the determination of the three-dimensional structure of the antigen-antibody complex by X-ray crystallography. This technique is, however, not always easy to perform due to the difficulty of obtaining high concentrations of a good quality complex and finding the proper conditions of crystallisation [8, 38]. Alternative biophysical techniques include (i) H/D exchange experiments on the antigen-antibody complex coupled to proteolysis with pepsin and subsequent analysis of the digested fragments by mass spectrometry (deuterium exchange mass spectrometry) [39] and (ii) NMR spectroscopy by comparing, for example, *heteronuclear single quantum coherence* (HSQC) spectra, of small target proteins in the presence or absence of the antibodies [40]. For all these structural approaches, high quantities of pure and stable antigens are however required, and some of them are limited by the size of the complex [8]. Another set of approaches is based on the exposition of numerous small peptides (overlapping sequences from the natural antigen or peptide mixtures derived from a combinatorial library if the antigen sequence is unknown) on a chip (peptide arrays) [41], or at the surface of phages (phage display) [42–46]. Phage display is based on the expression of a peptide/protein/protein fragment of interest at the surface of phage particles, fused to one of their coat proteins [42, 47, 48]. The power of this technique is the physical link between the phenotype (the expression of the peptide/protein/protein fragment of interest that can interact with its ligand) and the genotype (the nucleotide sequence of the peptide/protein/protein fragment cloned into the phagemid genome) [42, 48]. Phage display allows high-throughput screening of libraries of variant nucleotide sequences with diversity up to 10^6^ to 10^10^ [11, 42, 49]. 

Innovative phage display strategies are continuously implemented [50]. One of them is based on the use of the *β*-lactamase hybrid protein to expose random peptides/protein fragments at the surface of the phages and therefore to enzymatically functionalize the epitope (Figure 3) [8, 11, 51]. The advantages of this strategy are numerous [11, 51]. First, the polypeptide exposed within the *β*-lactamase could have a restricted conformational freedom and be somehow protected from proteolytic cleavage [3]. As illustrated in Figure 3, the main implementation is, however, associated with the use of *β*-lactamase activity which can be easily detected with chromogenic substrates such as nitrocefin [11]. The *β*-lactamase activity is used (i) as a reporter to directly assess the interactions between the inserted peptides and the target antibodies, and to easily monitor the enrichment of the phage library during the successive rounds of selection, and (ii) as an agent of selection of phages expressing active BHPs. Indeed, in order to amplify phages, phage-infected cells are grown in a liquid medium in the presence of ampicillin. Under these conditions, the bacterial growth is directly associated with antibiotic resistance, and thus only cells expressing active BlaP at the surface of phages are able to grow [11].

 This approach was first introduced by Legendre et al., who inserted random peptides within TEM-1, which was displayed on phage fd in fusion with the coat protein pIII [51]. The peptides were displayed on different loops surrounding the active site of TEM-1: in one library, peptides replaced residues A103 to 106; in a second library, they replaced residues Thr271 and/or Met272, and these two libraries were combined in a third one [51]. By selection from the different libraries using three unrelated conformational monoclonal antibodies (mabs) recognizing distinct epitopes on the prostate-specific antigen (PSA), several hybrid proteins expressing small peptides with an affinity for these mabs in the micro- and nanomolar range were isolated. The sequence of these small peptides presents no similarity with that of PSA, suggesting that mimotopes (i.e., peptides which bind the antibody without having any identity to the antigen sequence) were selected. These results indicate that BHPs could effectively be used to display peptides at the surface of phages. 

An original epitope mapping strategy, inspired by the work of Legendre et al., was developed by Bannister et al. and Chevigné et al. [8, 11]. It involves constructing a phage display library in which random fragments of different lengths of the gene coding for the antigen of interest are exposed within the *β*-lactamase BlaP (at position 197) in fusion with the pIII protein at the surface of phages (Figure 3). A given region of the target protein is displayed within peptides of different lengths and could therefore adopt different conformations. Sufficiently long peptides are likely to adopt a fold similar to what they adopt in the full target protein [11]. As exemplified below, this technology allows the minimal region of an antigen interacting with an antibody to be identified with high accuracy (Figure 3) [11]. As the peptides exposed within the *β*-lactamase are directly related to the nucleotide sequence of the antigen, they do not correspond to mimotopes. Moreover, the key amino acids within this minimal region that are directly in contact with the antibody can be further determined by point mutations as discussed below (Figure 3) [8]. 

### 4.1. Mapping of Linear Epitopes

The BHP-implemented phage display approach, developed by Chevigné et al. [11], has allowed the determination of the linear epitope (i.e., an epitope composed of amino acids that are in close proximity in the sequence) of a high-affinity monoclonal antibody (anti-*HA* mab) specific to the virus influenza hemagglutinin (HA1). Overlapping peptides of different sizes (from gene fragments of 50 to 300 bp) of HA1 were displayed on the solvent exposed loop between *α* helices 8 and 9 of BlaP, which was fused to pIII coat protein of phages (Figure 3). The phages expressing peptides containing the epitope region of HA1 were selected by panning against anti-*HA* mab. After three rounds of selection and amplification in the presence of ampicillin, a series of phages expressing BHPs specific to anti-*HA* mab was selected. The sequencing of these phages shows a consensus 9-residues linear epitope of anti-*HA* mab (Figure 4). This epitope is present in fragments of various sizes (from 13 to 70 residues) and can thus in principle adopt different folds and solvent accessibilities. The gene coding for the BHP displaying the consensus 9-residues epitope sequence was cloned into the constitutive expression vector pNY. The hybrid protein, referred to as BlaP-HA, was subsequently expressed in the periplasm of *E. coli* and purified as a bifunctional hybrid protein. The kinetic parameters (i.e., *K*_*m*_, *k*_cat_, and *k*_cat_/*K*_*m*_) of BlaP-HA are similar to that of wild-type BlaP, and it binds anti-*HA* mab with an affinity (*K*_*D*_) of ~0.68 nM (Table 1) [11]. 

### 4.2. Mapping of Conformational Epitopes

A similar approach was used by Bannister et al. to identify the conformational epitope (i.e., epitope composed of amino acids located far apart in the sequence but brought together by protein folding) of the anti-CD22 immunotoxin CAT-8015 (mab 8015) [8]. CD22 (cluster of differentiation-22) is a cell surface glycoprotein composed of a N-terminal Ig-like V-type domain and various Ig-like C-type domains (Figure 5) [52–55]. This protein is of particular therapeutic interest because it is a specific marker present on the surface of malignant B-cells and it is rapidly internalized upon binding; it constitutes therefore a relevant target for an antibody drug conjugate or immunotoxin approach. Despite the therapeutic interest of CD22, very little is known concerning its structure or that of the other related family members due to their high level of glycosylation [8]. CAT-8015 is an immunotoxin which combines a CD22-specific antibody variable fragment (Fv, derived from the antibody mab 8015) with a *Pseudomonas* exotoxin A (PE38); it exhibits a noteworthy clinical activity in three leukaemia (i.e., chronic lymphocyte leukaemia, hairy cell leukaemia, and acute lymphoblastic leukaemia) [8, 56, 57]. Antibody competition-binding studies have revealed that the epitope of CAT-8015 is localized in the C-like domain 2 of CD22, but there is no information on its precise location [8, 58]. 

In order to identify which residues of CD22 bind to CAT-8015, Bannister et al. introduced random CD22 extracellular domain gene fragments of 50 to 1000 bp into the permissive exposed loop of BlaP (position 197) fused to the phage pIII coat protein (Figure 3) [8]. A library containing 6 × 10^5^ transformants was obtained and screened against CAT-8015 using the same strategy as that explained above. A peptide-array analysis (Figure 3) confirmed that the entire CD22 gene was well represented in the *β*-lactamase-positive infectious phages, except two small regions of 7 residues each. The minimal region of CD22 which binds to mab 8015 was identified. This region, referred to as CD22/C2C3, is composed of 202 residues, from V234 to G435, located in the C-terminal of the C-type domain 1, in the C-type domains 2 and 3, and in the N-terminal of the C-type domain 4 (Figure 5).

The gene coding for the BHP displaying the minimal region of CD22 was cloned into the constitutive expression vector pNY. The hybrid BlaP-CD22/C2C3, produced as a bifunctional hybrid protein in *E. coli*, conserves the *β*-lactamase activity and binds to mab 8015 with a high affinity (*K*_*D*_ ~26.2 nM) (Table 1). To identify the key amino acids involved in the antibody binding, an alanine-scanning mutagenesis was performed (Figure 3) [11]. Thirty-four single-point mutations to alanine were performed in three clusters (referred to as clusters 1, 2, and 3) of CD22 encompassing the epitope, and the resulting hybrid proteins were produced and purified. Cluster 1 is located in the junction of C-type domains 1 and 2, cluster 2 is located in C-type domain 3 and cluster 3 encompasses the junction between C-type domain 3 and 4 and the N-terminal of C-type domain 4 (Figure 5). The binding of each mutant to mab 8015 was then measured by enzyme-linked immunosorbent assay (ELISA) and compared to that of the parent hybrid protein BlaP-CD22/C2C3. This technique has allowed the identification of the amino acids of high or intermediate importance in the CD22-mab 8015 complex. The most important residues encompass three discontinuous regions and they are mainly located in C-type domains 2 and 3 (clusters 1 and 2), and few are located in cluster 3. Modelling of different orientations of these domains strongly suggests that they adopt a U-shaped arrangement which allows the three clusters to be in close enough proximity to form the epitope (Figure 5) [8].

 These two examples show that alternating successive affinity selections of phages and growth of phage-infected cells in the presence of antibiotic permits the selection of BHPs exhibiting both a high affinity for the target antigen and an efficient enzymatic activity. They clearly demonstrate that BHP technology using BlaP is a unique tool that allows the identification of the antigen region involved in the antigen-antibody interactions. It allows (i) the identification of linear epitopes (i.e., the linear epitope of HA for anti-*HA* mab) and (ii) the characterisation of complex epitopes (i.e., the U-shaped discontinuous CD22 epitope of mab 8015). Moreover, BlaP has enough conformational flexibility to allow inserted antigen fragments of various lengths to fold and interact with the antibody. BHPs allow therefore the identification of non-linear epitopes (i.e., conformational epitopes) that are directly linked to the nucleotide sequence of the antigen (i.e., not a mimotope) [8, 11]. This approach can be further used to identify the protein region involved in any protein-ligand interactions. 

### 4.3. BHPs as a Unique Tool for Immunoassay Development

The *β*-lactamase implemented phage-display technique described above allows the selection of a particular epitope as a bifunctional hybrid protein which associates the epitope recognizing its specific target with an efficient enzymatic activity. This functionalization of the epitope allows the rapid characterisation of the antigen-antibody interaction. For example, the BlaP-HA hybrid protein was successfully coated on solid surface to perform an ELISA, suggesting that the solvent accessibility of the inserted polypeptide (i.e., the epitope) was not altered when the hybrid protein is coated [11]. Moreover, the enzymatic activity of BlaP can be used to check the coating efficiency and to quantify the amount of coated protein.

## 5. BHPs as Immunogenic Carriers for Vaccine Development

Antibodies are specialized fighter proteins that are effective in preventing infectious diseases. This property is based on the recognition of specific epitopes on the surface of the antigen that promotes the neutralization of the biological activity of the antigen or the opsonisation of the pathological agent. It is assumed that immunization with a precise epitope, corresponding to an effective neutralizing antibody, would elicit the generation of similarly potent antibodies in the vaccine [38]. Thus, the insertion of these particular epitopes into a carrier protein is often the starting point for the development of a new generation of safe vaccines. Within the carrier protein, the properties of the polypeptides, including their antigenicity and immunogenicity, can be further modified [59]. In this context, the BHP technology, allowing the insertion of a domain, subdomain, or a short polypeptide from the native targeted antigen into a carrier *β*-lactamase, is of particular interest to design such *de novo* antigens (Figure 6). This approach is particularly relevant to antibody raised against cryptic epitopes and non-immunodominant antigens.

### 5.1. Generation of Vaccines against Poorly Immunogenic Polypeptides/Proteins

TEM-1 hybrid proteins were created in an attempt to develop a vaccine against the poorly antigenic and non-immunogenic STa enterotoxin from enterotoxic *E. coli *strains (ETEC). This toxin, which is associated with enteric colibacillosis (characterized by severe diarrhoea) in calves and piglets, leads to significant losses in agriculture due to the death of newborns [60, 61]. STa is composed of 18 amino acids including 6 cysteins involved in three disulfide bridges which are necessary for the toxic activity [62, 63]. STa is poorly antigenic and is not immunogenic due to its small size. No vaccine is yet available against this thermostable toxin despite many attempts to design a safe vaccine (i.e., a non-toxic form of STa). The latter includes the chemical coupling of the toxin to bovine serum albumin [64, 65], to the *β*-subunit of cholera toxin [66], and to the heat-labile enterotoxin (LT) [65, 67], and its fusion to the major protein subunit ClpG of *E. coli* CS31A surface antigen [68], to several subunits of cholera toxin [66, 69], to LT [70, 71], to OmpC [70], and to flagellin [72]. These constructions either failed to induce the production of neutralizing antibodies against STa or retained a certain degree of toxicity. However, Wu and Chung have managed to elicit the production of protective antibodies against the antigen STLT (i.e., a fusion of the thermostable ST and thermolabile LT enterotoxins) in mice using a protein fusion between GFP and STLT. These immunized mice presented a subsequent full protection against ETEC [73].

Different approaches based on the use of TEM-1 hybrid proteins have been used in order to design a vaccine against STa [9, 14, 15]. First, Ruth et al. have designed DNA vaccination to induce the production of neutralizing antibodies against STa [14]. STa and three variant forms, in which one (STaC6A, STaC17A) or two (STaC6A-C17A) of the six cysteines have been mutated (in order to disrupt one or two disulphide bridges and cause a complete loss of the toxicity of the toxin), have been inserted either in position 195 (loop A) or 216 (loop B) of TEM-1. Plasmid DNA encoding these hybrid proteins has been used to immunize mice. Following immunizations, different levels of anti TEM-1 antibodies were generated. The level of antibody production against TEM-1 was higher for mice immunized with plasmid DNA coding for BHPs displaying STa and its variants in position 216 (loop B) than in position 195 (loop A). Since insertions in loop B interfere less with anti TEM-1 antibody production than insertion in loop A, this suggests that the immunodominant epitope of TEM-1 is located in the region of loop A. In contrast, no antibody specific to STa could be detected, even after 3 injections of the different plasmids. Two subsequent boosts with a STa toxin obtained by peptide synthesis, which is not immunogenic, did however induce the production of STa-specific antibodies in mice initially primed with plasmids encoding hybrid proteins, but not when primed with plasmid encoding TEM-1. This clearly indicates that hybrid proteins were expressed in mice and have primed the production of antibodies specific to STa. The ability of sera containing STa specific antibodies to neutralize the toxin was determined by suckling mouse assays. Only the sera from mice immunized with the plasmid coding for the double disulfide bridge mutated variant (STaC6A-C17A) and boosted with STa injections show neutralizing activity. These results indicate that the use of the toxic form of STa is therefore not needed to induce the production of neutralizing antibodies. These results also indicate that TEM-1 is an appropriate carrier to present nonimmunogenic peptide to the immune system. Indeed, the carrier is required for the induction of helper T cells allowing the production of antibodies against the carrier, TEM-1, and the hapten, STa. Moreover, the best location for the insertion seems to be located at position 195, the immunodominant epitope of TEM-1. Indeed, exposing the insert at this position reduces the production of anti TEM-1 antibodies and should therefore decrease the competition between the hapten and the carrier for the B-cell immune response [14].

Subsequently, recombinant hybrid TEM-1 proteins in which STa has been inserted at different positions, including positions 195 and 216, were designed, produced, and used for mice immunization (Figure 6) [9]. This study revealed that the hybrid proteins elicit the production of antibodies mainly against TEM-1, and in much lower quantity against STa. TEM-1 with the insertion at position 195 induces the highest production of anti-STa antibody and most importantly was the only hybrid protein that leads to the production of antibodies neutralizing the toxicity of STa. These results are in good agreement with results obtained with DNA vaccination and confirm that B-cell epitopes of the carrier are immunodominant. Moreover, the carrier, TEM-1, contains the functional helper T cell epitopes necessary for the immune response against the hapten, STa [9]. 

Following these encouraging results, Zervosen et al. immunized cattle with a TEM-1 hybrid protein containing the STa in position 197 in the presence of 3 different adjuvants (Table 1) (Montanide ISA70 - ISA206 and IMS1313) [15]. High levels of different IgG types specific to TEM-1 were detected, and *in vitro* neutralization of the *β*-lactamase activity was observed by mixing purified TEM-1 with sera. In contrast, specific anti-STa IgG and IgG1 antibodies were only detected at non-significant levels, and no IgG2 were detected in the sera of the immunized cattle. These results suggest that the response of the bovine immune system is different from that observed in mice [9, 15]. The use of a series of other adjuvants to immunize cattle needs to be investigated.

### 5.2. Production of Neutralizing Antibodies against Difficult-to-Express Antigens

As discussed above, BlaP can be used as a scaffold to produce and to purify the chitin binding domain from chitotriosidase (ChBD) [13]. The purified ChBD has been used to immunize a rabbit (Figure 6). The resulting serum contains antibodies that are able to bind to the free ChBD, the hybrid BlaP-*Thb/ChBD/Thb*, and the native human macrophage chitotriosidase. Moreover, these anti-ChBD antibodies are able to prevent the interaction of ChBD with chitin [13]. 

Taken all together, the results of these studies indicate that both BlaP and TEM-1 are appropriate scaffolds for producing and presenting antigens and inducing the production of antibodies neutralizing biological properties of the inserted fragment (Figure 6).

## 6. BHPs as Model Proteins to Investigate Structure/Function Relationships 

### 6.1. BlaP: A Scaffold to Create Protein Models to Study the Mechanism of Amyloid Fibril Formation by Polyglutamine Proteins

Ten progressive neurodegenerative disorders, referred to as polyglutamine (polyQ) diseases, and, including Huntington's disease and several spinocerebellar ataxias, are associated with ten unrelated proteins containing an expanded polyglutamine (polyQ) tract (i.e., a tract that is longer than a pathological polyglutamine threshold). PolyQ tracts are encoded by a repetition of an unstable CAG trinucleotide repeat in the corresponding genes [74–77]. The ten disease-associated proteins show no sequence or structural similarity apart from the expanded polyQ tract, which is located at a different positions in each protein. The polyQ tract appears therefore to be a critical determinant in polyQ diseases, and several lines of evidence suggest that it confers a gain of toxic function to the mutant proteins by triggering the aggregation of the proteins into amyloid fibrils [74, 75, 78–80]. Indeed, all polyQ diseases share a number of features which suggest a common physiopathological mechanism [75, 79–81]: (i) the existence of a polyQ threshold for the aggregation of polyQ proteins and the disease development, generally comprised between 35 and 45Q [82], (ii) the so-called anticipation phenomenon, which indicates that the longer the polyQ, the earlier and more severe the disease [76, 83–85], and (iii) the presence of intranuclear inclusion bodies, containing amyloid fibrils made of polyQ proteins, in neuronal cells [75, 76, 85, 86]. 

So far, there is no preventive or curative treatment for these pathologies and existing therapies only treat the symptoms (i.e., they alleviate the symptoms without modifying the course of the disease). In order to design curative and/or preventive treatments, it is crucial to better understand how polyQ tracts trigger protein aggregation and by which mechanism some of the aggregates formed are cytotoxic. 

Although the presence of the expanded polyQ tract is the critical trigger factor of the aggregation phenomenon, a growing number of studies suggest that the non-polyQ regions can, however, modulate both the kinetics and the aggregation pathway of polyQ proteins [74, 78, 87–90]. The non-polyQ regions can protect from aggregation by (i) sterically hindering polyQ intermolecular interactions [91], (ii) restricting polyQ conformational changes which are required for fibril formation [89] and (iii) increasing the protein solubility [87, 91]. On the other hand, non-polyQ regions could assist aggregation by providing additional aggregation-prone domains [74, 92]. There is, therefore, a complex interplay between the tendency of the polyQ tract to trigger aggregation and the modulating effect of non-polyQ regions [16]. To better understand the general principles governing this complex phenomenon, it is crucial to investigate in detail which properties of the host protein (sequence, size, structure, and stability) influence the ability of polyQ tracts to mediate aggregation. The ten disease-associated proteins are difficult to produce recombinantly due to their large size and/or relative insolubility [74, 92–94]. Scarafone et al. tackled this problem by creating and characterizing model polyQ proteins consisting of the *β*-lactamase BlaP and polyQ tracts inserted at position 197 [16]. Significant amounts (i.e., 10–20 mg per liter of culture) of hybrid enzymes containing 23, 30, 55, and 79Q were successfully produced and purified. It is important to note that the longest polyQ tract that has been inserted in other model proteins is made of 55 residues [95]. BlaP is therefore a unique scaffold to investigate the effects of long inserted polyQ sequences (Figure 7).

The effects of the polyQ insertions on the activity, structure, and aggregation of BlaP were investigated using a range of biophysical techniques. The activity and the secondary and tertiary structures of BlaP are essentially not affected by the insertion of the polyQ tract as long as 79Q. The polyQ tract adopts a disordered structure at the surface of the protein irrespective of the number of glutamines. BlaP is significantly destabilized, however, by the insertion of the polyQ tract. Remarkably, the extent of destabilization is largely independent of the polyQ length (7.6–8.8 kJ·mol^−1^; Table 1). This behaviour therefore makes it possible to investigate independently the role of (i) the length of the polyQ sequence and (ii) the conformational state of the *β*-lactamase moiety on the aggregating properties of the hybrid proteins. Accordingly, the aggregating properties of BlaP and of the different hybrid proteins were investigated under both native and denaturing conditions. The aggregation behaviour of BlaP-polyQ hybrid proteins recapitulates that of disease-associated polyQ proteins. Only hybrid proteins with 55Q and 79Q readily form amyloid fibrils; therefore, analogous to the proteins associated with diseases, there is a polyglutamine threshold required for the formation of amyloid fibrils. Moreover, above this threshold, the longer the polyQ, the faster the aggregation rate (Figure 7). Most importantly, the threshold-value critically depends on the structural integrity of BlaP. BlaP with 55Q forms fibrils under denaturing but not under native conditions (Figure 7). This means that the native conformation of BlaP imposes some conformational and/or steric constraints to the 55Q tract that inhibit fibril formation. On the other hand, the hybrid protein containing 79Q forms amyloid fibrils at similar rates whether BlaP is folded or not (Figure 7). These results therefore suggest that the influence of the protein context on the aggregation properties of polyQ disease-associated proteins could be negligible when the latter contain particularly long polyQ tracts [16]. 

Taken all together, these results indicate that BlaP is an appropriate host to study the aggregation of polyQ proteins. Its utility could be extended to the study of how other amyloidogenic peptides trigger protein aggregation.

### 6.2. Effect of the Structure of the Insert on BHP Stabilities

Vandevenne et al. [10] extensively investigated the effects of the insertion of the ChBD domain on the thermodynamic stability of BlaP, as indicated above. They observed that the insertion of this 72-residue folded domain at position 197 slightly destabilizes BlaP by 3.2 kJ·mol^−1^ (Table 1) [10]. This destabilization is significantly lower than that induced by the insertion of unstructured polyQ tracts of 23 to 79 residues, inserted into the same position (7.6–8.8 kJ·mol^−1^, Table 1) [16]. This observation suggests that the insertion of unstructured polypeptides is more destabilizing than the insertion of folded polypeptides.

### 6.3. BHPs as Models to Screen Molecules Stabilizing Polypeptides

 A growing number of peptide and protein drugs are utilized in therapy [96]. Unfortunately, because of unfavourable solubility, stability, and aggregation, their applications are sometimes difficult [96]. To circumvent this problem, low molecular weight additives, called cosolutes, have been developed, including cyclodextrins [96, 97]. Cyclodextrins are circular oligosaccharides containing a central cavity forming the resting site for hydrophobic molecules of an appropriate dimension [98]. They are generally used to prevent protein aggregation during the renaturation process [12, 96]. BCD07056 is a modified *β*-cyclodextrin, one of the most abundant classes of cyclodextrin [96]. 

 Vandevenne et al. used the hybrid protein BlaP-ChBD, incubated under drastic conditions, to investigate the effects of BCD07056 on the stability of proteins [12]. They observed that BCD07056 does not affect the chitin binding of BlaP-ChBD, yet increases its *β*-lactamase activity. More interestingly, this *β*-cyclodextrin minimizes the inactivation of BlaP-ChBD upon storage at room temperature; its addition cannot, however, reverse the inactivation process. The *β*-cyclodextrin has a moderate effect on the thermal stability of BlaP-ChBD. However, its presence restores a cooperative reversible thermal unfolding, with a simple two-state transition, characteristic of BlaP without insert. This suggests that BCD07056 prevents the aggregation of BlaP-ChBD by interacting with the protein during the unfolding process. BCD07056 is therefore an effective additive to stabilize proteins during their storage and prevent their aggregation, without interfering with their activity [12]. It could be used to facilitate the application of a growing number of peptide and protein drugs in therapy [96].

## 7. Conclusion

Class A *β*-lactamase hybrid proteins, in which exogenous polypeptides of various sizes are inserted (up to 40 kDa), can be readily designed and used for multiple purposes, notably to produce difficult-to-express peptides/proteins/protein fragments, to map epitopes, to display antigens, and to study protein structure/function relationships. The wide ranging impact of the BHP approach essentially originates from (i) the efficient enzymatic activity that can be easily measured and that can serve as a reporter or factor for selection and (ii) the facility with which they can be recombinantly produced and purified. In addition to the numerous applications summarized in this review, many other applications can be envisaged: BHPs could be used as biosensors and in affinity chromatography, drug screening, and drug targeting. They are also of special interest to better understand more fundamental aspects of protein evolution and structure/function relationships.

## Figures and Tables

**Figure 1:** X-ray crystal structure and sequence of TEM-1 (a) and BlaP (b). The residue numbering is based on homology to class A *β*-lactamases [17]. The structures were produced using PyMOL (DeLano Scientific LLC, South San Francisco, CA, USA) and the PDB ID is 4BLM for BlaP [18] and 1XPB for TEM-1 [19]. (a) TEM-1. The residues of the active site are represented in green on the structure and are coloured and underlined in the sequence. The different insertion sites of pentapeptides reported in Hallet et al. [20] are coloured on the structure and are coloured and underlined in the sequence. Light blue, orange and red are associated with permissive, semi-permissive, and non-permissive insertion sites, respectively. (b) BlaP from *Bacillus licheniformis* 749/C. The residues of the active site are represented in green on the structure, and are coloured and underlined in the sequence. The two insertion sites most commonly used to design BHPs, located in the loop between *α* helices 8 and 9 (197-198) and in the loop between *α* helices 9 and 10 (216-217), are indicated in light blue on the structure and are coloured and underlined in the sequence. The PG dipeptide between residues 197 and 198 indicated in bold in the sequence corresponds to the SmaI restriction site inserted into the gene of BlaP for the cloning of exogenous polypeptides at this position.

**Figure 2:** Schematic representation of the protocol used to cleave the ChBD domain from BlaP and to purify it. Purified ChBD is collected in the flow through after loading the hybrid protein digested by thrombin on an immobilized metal ion affinity chromatography (IMAC). Figure adapted from Vandevenne et al., 2008 [13]. BlaP-Cter: C-terminal sequence of BlaP, starting at the insertion site. BlaP-Nter: N-terminal sequence of BlaP ending at the insertion site.

**Figure 3:** BHPs as unique tools for epitope mapping. Schematic representation of the epitope mapping procedure developed by Bannister et al. and Chevigné et al. [8, 11]. The steps for which the enzymatic activity of BlaP, as a reporter or as factor for selection, is critical are highlighted in red. BlaP-Cter: C-terminal sequence of BlaP, starting at the insertion site. BlaP-Nter: N-terminal sequence of BlaP ending at the insertion site. Anti-Ag mab: monoclonal antibody specific to the targeted antigen. Following the elution of phages after the last round of panning, a peptide array can be carried out to verify that the entire antigen sequence is well represented in the phage library. Alanine scanning mutagenesis can be carried out to determine which residues of the minimal sequence encompassing the epitope is in direct contact with the antigen. Figure adapted from Chevigné et al., 2007 [11].

**Figure 4:** Consensus sequence recognized by anti-HA mab. Multiple sequence alignment from eleven individual clones selected after three rounds of selection of phages on anti-HA mab. The residues corresponding to the epitope recognized by the anti-HA mab are underlined. Figure from Chevigné et al. [11].

**Figure 5:** Schematic representations of the glycoprotein CD22 in a linear and U-shaped arrangement. In the linear arrangement, the three clusters forming the epitope are far away from each other whereas they are close in a U-shaped arrangement [8]. The residues involved in the complex with mab 8015 are clustered in cluster 1, 2, and 3 and are shown in light blue, red, and green, respectively. Figure adapted from Bannister et al. [8].

**Figure 6:** Schematic representation of the BHP technology used to design *de novo* antigens in order to induce the production of neutralizing antibodies. A specific region of a large antigen, that is known to promote the neutralization of the biological activity of the antigen or promote its opsonization, is inserted into BlaP. This approach can also be used to elicit the production of specific, neutralizing antibodies against polypeptides that are insoluble, difficult to express (i.e., ChBD, [13]), and poorly immunogenic (such as STa, [9]).

**Figure 7:** Model polyQ proteins using BlaP to investigate the amyloid fibril formation. The advantage of using BlaP as a scaffold to create polyQ proteins are highlighted in red. Left side panel: schematic representation of the polyQ-BlaP hybrid protein. Middle panel: kinetics of aggregation of BlaP_197_(Gln)_55_ and BlaP_197_(Gln)_79_ at 110 *μ*M under the following conditions of incubation: (i) PBS, pH 7.5 and 0 M urea at 37°C (pink), (ii) PBS, pH 7.5, and 1.85 M urea at 25°C (blue) and (iii) PBS, pH 7.5, and 3.5 M urea at 25°C (green). BlaP_197_(Gln)_55_ does not form amyloid fibrils under native conditions, in contrast to BlaP_197_(Gln)_79_. Under native conditions, the threshold value is therefore comprised between 55 and 79Q. Under denaturing conditions, it is comprised between 30 and 55Q. Moreover, the kinetics of aggregation are faster with longer polyQ tracts. Right side panel: schematic pathway of aggregation for BlaP_197_(Gln)_55_ and BlaP_197_(Gln)_79_. N, native state; U, unfolded state; F, amyloid fibril. The native conformation of BlaP imposes constraints to the 55Q tract that prevent it to trigger the formation of amyloid fibrils. Figure adapted from Scarafone et al. [16].

**Table 1:** Properties of the different BHPs discussed in this review.

Hybrid proteins [ref]	Insert		Effect on stability (ΔΔG_H_2_O_°—kJ·mol^−1^)	Effects on the *β*-lactamase activity	Function of the insert
	Name + size	Insertion site			
TEM-1-STa [14, 15]	STa 18 AA	37, 195, 197, 198, 206, 216, 218, 232 and 260	ND	Insertion at positions 37, 198, and 206: ND Insertion at position 195: no loss of activity Insertion at positions 197, 216, 232, and 260: partial loss of activity	Enterotoxicity

BlaP-HA [11]	HA 9 AA	197	ND	No loss of activity	Binding to anti-HA mab: *K*_*D*_ = 0.68 nM

BlaP-ChBD [10]	ChBD 72 AA	197	~3.2	No loss or partial loss of activity depending on the substrate	Binding to chitin: *K*_*r*_ = 5.4 ± 0.5 L g^−1^
	Thb-ChBD-Thb	197	ND	Partial loss of activity	Binding to chitin

BlaP-CD22 [12]	CD22/C2C3 202 AA	197	ND	Activity detected but not quantified	Binding to mab 8015: *K*_*D*_ = 26.2 ± 1.4 nM

BlaP_197_(Gln)_*x*_ [16]	PolyQ tracts 23Q-30Q-55Q and 79Q	197	~7.6–8.8	No loss of activity	PolyQ tracts longer than a threshold trigger the aggregation of BHPs into amyloid fibrils

The name of the BHPs, the name of the insert, its size, and function are indicated. The effects of the insertion on the stability and on the enzymatic activity of the *β*-lactamase are also reported. ND: not determined.

## Abbreviations

Ag: Antigen
BHPs: *β*-lactamase hybrid proteins
BlaP: *β*-lactamase from *Bacillus licheniformis* 749/C
CD22: Cluster of differentiation-22
ChBD: Chitin binding domain
dsbA: Disulfide bond isomerase A
ELISA: Enzyme-linked immunosorbent assay
ETEC: Enterotoxic *E. coli *
GFP: Green fluorescent protein
HA1: Virus influenza hemagglutinin
H/D: Hydrogen/deuterium
LT: Thermolabile enterotoxin
mab: Monoclonal antibody
MalE: Maltodextrin-binding protein
NMR: Nuclear magnetic resonance
polyQ: Polyglutamine
PSA: Prostate specific antigen
Thb: thrombin.

## References

[1] Beguin P (1999). Hybrid enzymes. *Current Opinion in Biotechnology*.

[2] Collinet B, Hervé M, Pecorari F, Minard P, Eder O, Desmadril M (2000). Functionally accepted insertions of proteins within protein domains. *Journal of Biological Chemistry*.

[3] Betton J-M, Jacob JP, Hofnung M, Broome-Smith JK (1997). Creating a bifunctional protein by insertion of *β*-lactamase into the maltodextrin-binding protein. *Nature Biotechnology*.

[4] Martin JL, Bardwell JCA, Kuriyan J (1993). Crystal structure of the DsbA protein required for disulphide bond formation in vivo. *Nature*.

[5] Delarue M, Poch O, Tordo N, Moras D, Argos P (1990). An attempt to unify the structure of polymerases. *Protein Engineering*.

[6] Levine M, Muirhead H, Stammers DK, Stuart DI (1978). Structure of pyruvate kinase and similarities with other enzymes: possible implications for protein taxonomy and evolution. *Nature*.

[7] Jones S, Stewart M, Michie A, Swindells MB, Orengo C, Thornton JM (1998). Domain assignment for protein structures using a consensus approach: characterization and analysis. *Protein Science*.

[8] Bannister D, Popovic B, Sridharan S (2011). Epitope mapping and key amino acid identification of anti-CD22 immunotoxin CAT-8015 using hybrid-lactamase display. *Protein Engineering, Design and Selection*.

[9] Ruth N, Quinting B, Mainil J (2008). Creating hybrid proteins by insertion of exogenous peptides into permissive sites of a class A *β*-lactamase. *FEBS Journal*.

[10] Vandevenne M, Filee P, Scarafone N (2007). The Bacillus licheniformis BlaP *β*-lactamase as a model protein scaffold to study the insertion of protein fragments. *Protein Science*.

[11] Chevigné A, Yilmaz N, Gaspard G (2007). Use of bifunctional hybrid *β*-lactamases for epitope mapping and immunoassay development. *Journal of Immunological Methods*.

[12] Vandevenne M, Gaspard G, Belgsir EM (2011). Effects of monopropanediamino-*β*-cyclodextrin on the denaturation process of the hybrid protein BlaPChBD. *Biochimica et Biophysica Acta*.

[13] Vandevenne M, Gaspard G, Yilmaz N (2008). Rapid and easy development of versatile tools to study protein/ligand interactions. *Protein Engineering, Design and Selection*.

[14] Ruth N, Mainil J, Roupie V, Frère J-M, Galleni M, Huygen K (2005). DNA vaccination for the priming of neutralizing antibodies against non-immunogenic STa enterotoxin from enterotoxigenic *Escherichia coli*. *Vaccine*.

[15] Zervosen A, Saegerman C, Antoniotti I (2008). Characterization of the cattle serum antibody responses against TEM *β*-lactamase and the nonimmunogenic *Escherichia coli* heat-stable enterotoxin (STaI). *FEMS Immunology and Medical Microbiology*.

[16] Scarafone N, Pain C, Fratamico A (2012). Amyloid-like fibril formation by polyq proteins: a critical balance between the polyq length and the constraints imposed by the host protein. *PLoS One*.

[17] Ambler RP, Coulson AFW, Frere J-M (1991). A standard numbering scheme for the class A *β*-lactamases. *Biochemical Journal*.

[18] Knox JR, Moews PC (1991). -Lactamase of Bacillus licheniformis 749/C. Refinement at 2 Å resolution and analysis of hydration. *Journal of Molecular Biology*.

[19] Fonze E, Charlier P, To’th Y (1995). TEM1 beta-lactamase structure solved by molecular replacement and refined structure of the S235A mutant. *Acta Crystallographica D*.

[20] Hallet B, Sherratt DJ, Hayes F (1997). Pentapeptide scanning mutagenesis: random insertion of a variable five amino acid cassette in a target protein. *Nucleic Acids Research*.

[21] Moore JT, Davis ST, Dev IK (1997). The development of *β*-lactamase as a highly versatile genetic reporter for eukaryotic cells. *Analytical Biochemistry*.

[22] Zlokarnik G, Negulescu PA, Knapp TE (1998). Quantitation of transcription and clonal selection of single living cells with *β*-lactamase as reporter. *Science*.

[23] Oosterom J, van Doornmalen EJP, Lobregt S, Blomenröhr M, Zaman GJR (2005). High-throughput screening using *β*-lactamase reporter-gene technology for identification of low-molecular-weight antagonists of the human gonadotropin releasing hormone receptor. *Assay and Drug Development Technologies*.

[24] Vandevenne M, Galleni M, Filee P (2011). How to make a good use of a “Bad Enzyme”: utilisation of efficient beta-lactamase for the benefits of biochemical research. *Beta-Lactamases*.

[25] Jelsch C, Mourey L, Masson J-M, Samama J-P (1993). Crystal structure of *Escherichia coli* TEM1 *β*-lactamase at 1.8 Å resolution. *Proteins*.

[26] Moews PC, Knox JR, Dideberg O, Charlier P, Frere J-M (1990). *β*-Lactamase of Bacillus licheniformis 749/C at 2 Å resolution. *Proteins*.

[27] Charpentier X, Oswald E (2004). Identification of the secretion and translocation domain of the enteropathogenic and enterohemorrhagic *Escherichia coli* effector Cif, using TEM-1 *β*-lactamase as a new fluorescence-based reporter. *Journal of Bacteriology*.

[28] Matagne A, Misselyn-Bauduin A-M, Joris B, Erpicum T, Granier B, Frere J-M (1990). The diversity of the catalytic properties of class A *β*-lactamases. *Biochemical Journal*.

[29] Wu X-C, Lee W, Tran L, Wong S-L (1991). Engineering a Bacillus subtilis expression-secretion system with a strain deficient in six extracellular proteases. *Journal of Bacteriology*.

[30] Veith B, Herzberg C, Steckel S (2004). The complete genome sequence of Bacillus licheniformis DSM13, an organism with great industrial potential. *Journal of Molecular Microbiology and Biotechnology*.

[31] Tjoelker LW, Gosting L, Frey S (2000). Structural and functional definition of the human chitinase chitin- binding domain. *Journal of Biological Chemistry*.

[32] Hollak CEM, Van Weely S, Van Oers MHJ, Aerts JMFG (1994). Marked elevation of plasma chitotriosidase activity. A novel hallmark of Gaucher disease. *Journal of Clinical Investigation*.

[33] Boot RG, Van Achterberg TAE, Van Aken BE (1999). Strong induction of members of the chitinase family of proteins in atherosclerosis: chitotriosidase and human cartilage gp-39 expressed in lesion macrophages. *Arteriosclerosis, Thrombosis, and Vascular Biology*.

[34] Overdijk B, Van Steijn GJ (1994). Human serum contains a chitinase: identification of an enzyme, formerly described as 4-metbylumbelliferyl-tetra-N-acetylchitotetraoside hydrolase (MU-TACT hydrolase). *Glycobiology*.

[35] Overdijk B, Van Steijn GJ, Odds FC (1996). Chitinase levels in guinea pig blood are increased after systemic infection with *Aspergillus fumigatus*. *Glycobiology*.

[36] Dumoulin M, Last AM, Desmyter A (2003). A camelid antibody fragment inhibits the formation of amyloid fibrils by human lysozyme. *Nature*.

[37] De Genst E, Chan P, Pardon E A nanobody binding to non-amyloidogenic regions of the protein human lysozyme enhances partial unfolding but inhibits amyloid fibril formation.

[38] Gershoni JM, Roitburd-Berman A, Siman-Tov DD, Freund NT, Weiss Y (2007). Epitope mapping: the first step in developing epitope-based vaccines. *BioDrugs*.

[39] Obungu VH, Gelfanova V, Rathnachalam R, Bailey A, Sloan-Lancaster J, Huang L (2009). Determination of the mechanism of action of anti-FasL antibody by epitope mapping and homology modeling. *Biochemistry*.

[40] Paterson Y, Englander SW, Roder H (1990). An antibody binding site on cytochrome c defined by hydrogen exchange and two-dimensional NMR. *Science*.

[41] Reineke U, Volkmer-Engert R, Schneider-Mergener J (2001). Applications of peptide arrays prepared by the spot-technology. *Current Opinion in Biotechnology*.

[42] Smith GP, Scott JK (1993). Libraries of peptides and proteins displayed on filamentous phage. *Methods in Enzymology*.

[43] Zwick MB, Shen J, Scott JK (1998). Phage-displayed peptide libraries. *Current Opinion in Biotechnology*.

[44] Williams SC, Badley RA, Davis PJ, Puijk WC, Meloen RH (1998). Identification of epitopes within beta lactoglobulin recognised by polyclonal antibodies using phage display and PEPSCAN. *Journal of Immunological Methods*.

[45] Van Zonneveld A-J (1995). Identification of functional interaction sites on proteins using bacteriophage-displayed random epitope libraries. *Gene*.

[46] Wang L-F, Du Plessis DH, White JR, Hyatt AD, Eaton BT (1995). Use of a gene-targeted phage display random epitope library to map an antigenic determinant on the bluetongue virus outer capsid protein VP5. *Journal of Immunological Methods*.

[47] Smith GP (1985). Filamentous fusion phage: novel expression vectors that display cloned antigens on the virion surface. *Science*.

[48] Rodi DJ, Makowski L (1999). Phage-display technology—finding a needle in a vast molecular haystack. *Current Opinion in Biotechnology*.

[49] Clackson T, Hoogenboom HR, Griffiths AD, Winter G (1991). Making antibody fragments using phage display libraries. *Nature*.

[50] Pande J, Szewczyk MM, Grover AK (2010). Phage display: concept, innovations, applications and future. *Biotechnology Advances*.

[51] Legendre D, Soumillion P, Fastrez J (1999). Engineering a regulatable enzyme for homogeneous immunoassays. *Nature Biotechnology*.

[52] Du X, Beers R, FitzGerald DJ, Pastan I (2008). Differential cellular internalization of anti-CD19 and -CD22 immunotoxins results in different cytotoxic activity. *Cancer Research*.

[53] Clark EA (1993). CD22, a B cell-specific receptor, mediates adhesion and signal transduction. *Journal of Immunology*.

[54] Crocker PR, Varki A (2001). Siglecs, sialic acids and innate immunity. *Trends in Immunology*.

[55] May AP, Robinson RC, Vinson M, Crocker PR, Jones EY (1998). Crystal structure of the N-terminal domain of sialoadhesin in complex with 3′ sialyllactose at 1.85 Å resolution. *Molecular Cell*.

[56] Mussai F, Campana D, Bhojwani D (2010). Cytotoxicity of the anti-CD22 immunotoxin HA22 (CAT-8015) against paediatric acute lymphoblastic leukaemia: research paper. *British Journal of Haematology*.

[57] Alderson RF, Kreitman RJ, Chen T (2009). CAT-8015: a second-generation pseudomonas exotoxin a-based immunotherapy targeting CD22-expressing hematologic malignancies. *Clinical Cancer Research*.

[58] DiJoseph JF, Popplewell A, Tickle S (2005). Antibody-targeted chemotherapy of B-cell lymphoma using calicheamicin conjugated to murine or humanized antibody against CD22. *Cancer Immunology, Immunotherapy*.

[59] Leclerc C, Lo-Man R, Charbit A, Martineau P, Clement JM, Hofnung M (1994). Immunogenicity of viral B- and T-cell epitopes expressed in recombinant bacterial proteins. *International Reviews of Immunology*.

[60] Holland RE (1990). Some infectious causes of diarrhea in young farm animals. *Clinical Microbiology Reviews*.

[61] Nagy B, Fekete PZ (1999). Enterotoxigenic *Escherichia coli* (ETEC) in farm animals. *Veterinary Research*.

[62] Gariépy J, Judd AK, Schoolnik GK (1987). Importance of disulfide bridges in the structure and activity of *Escherichia coli* enterotoxin ST1b. *Proceedings of the National Academy of Sciences of the United States of America*.

[63] Moseley SL, Hardy JW, Huq MI (1983). Isolation and nucleotide sequence determination of a gene encoding a heat-stable enterotoxin of *Escherichia coli*. *Infection and Immunity*.

[64] Lockwood DE, Robertson DC (1984). Development of a competitive enzyme-linked immunosorbent assay (ELISA) for *Escherichia coli* heat-stable enterotoxin (ST(a)). *Journal of Immunological Methods*.

[65] Svennerholm A-M, Wikstrom M, Lindblad M, Holmgren J (1986). Monoclonal antibodies against *Escherichia coli* heat-stable toxin (STa) and their use in a diagnostic ST ganglioside GM1-enzyme-linked immunosorbent assay. *Journal of Clinical Microbiology*.

[66] Sanchez J, Svennerholm A-M, Holmgren J (1988). Genetic fusion of a non-toxic heat-stable enterotoxin-related decapeptide antigen to cholera toxin B-subunit. *FEBS Letters*.

[67] Klipstein FA, Engert RF, Clements JD, Houghten RA (1983). Vaccine for enterotoxigenic *Escherichia coli* based on synthetic heat-stable toxin crossed-linked to the B subunit of heat-labile toxin. *Journal of Infectious Diseases*.

[68] Batisson I, Der Vartanian M (2000). Contribution of defined amino acid residues to the immunogenicity of recombinant *Escherichia coli* heat-stable enterotoxin fusion proteins. *FEMS Microbiology Letters*.

[69] Sanchez J, Argotte R, Buelna A (1997). Engineering of cholera toxin A-subunit for carriage of epitopes at its amino end. *FEBS Letters*.

[70] Aitken R, Hirst TR (1993). Recombinant enterotoxins as vaccines against *Escherichia coli*-mediated diarrhoea. *Vaccine*.

[71] Sanchez J, Uhlin BE, Grundstrom T (1986). Immunoactive chimeric ST-LT enterotoxins of *Escherichia coli* generated by in vitro gene fusion. *FEBS Letters*.

[72] Pereira CM, Guth BE, Sbrogio-Almeida ME, Castilho BA (2001). Antibody response against *Escherichia coli* heat-stable enterotoxin expressed as fusions to flagellin. *Microbiology*.

[73] Wu C-M, Chung T-C (2007). Mice protected by oral immunization with Lactobacillus reuteri secreting fusion protein of *Escherichia coli* enterotoxin subunit protein. *FEMS Immunology and Medical Microbiology*.

[74] Hands SL, Wyttenbach A (2010). Neurotoxic protein oligomerisation associated with polyglutamine diseases. *Acta Neuropathologica*.

[75] Zoghbi HY, Orr HT (2000). Glutamine repeats and neurodegeneration. *Annual Review of Neuroscience*.

[76] Orr HT, Zoghbi HY (2007). Trinucleotide repeat disorders. *Annual Review of Neuroscience*.

[77] Ross CA (1997). Intranuclear neuronal inclusions: a common pathogenic mechanism for glutamine-repeat neurodegenerative diseases?. *Neuron*.

[78] Wetzel R, Alvarado MR, Kelly JW, Dobson CM (2010). Misfolding and aggregation in Huntington disease and other expanded Polyglutamine repeat diseases. *Protein Misfolding Diseases*.

[79] Ordway JM, Tallaksen-Greene S, Gutekunst C-A (1997). Ectopically expressed CAG repeats cause intranuclear inclusions and a progressive late onset neurological phenotype in the mouse. *Cell*.

[80] Chen YW, Stott K, Perutz MF (1999). Crystal structure of a dimeric chymotrypsin inhibitor 2 mutant containing an inserted glutamine repeat. *Proceedings of the National Academy of Sciences of the United States of America*.

[81] Gordon-Smith DJ, Carbajo RJ, Stott K, Neuhaus D (2001). Solution studies of chymotrypsin inhibitor-2 glutamine insertion mutants show no interglutamine interactions. *Biochemical and Biophysical Research Communications*.

[82] Ross CA (2002). Polyglutamine pathogenesis: emergence of unifying mechanisms for Huntington’s disease and related disorders. *Neuron*.

[83] Bauer PO, Nukina N (2009). The pathogenic mechanisms of polyglutamine diseases and current therapeutic strategies. *Journal of Neurochemistry*.

[84] Penney JB, Vonsattel J-P, MacDonald ME, Gusella JF, Myers RH (1997). CAG repeat number governs the development rate of pathology in huntington’s disease. *Annals of Neurology*.

[85] Schöls L, Bauer P, Schmidt T, Schulte T, Riess O (2004). Autosomal dominant cerebellar ataxias: clinical features, genetics, and pathogenesis. *Lancet Neurology*.

[86] Davies SW, Turmaine M, Cozens BA (1997). Formation of neuronal intranuclear inclusions underlies the neurological dysfunction in mice transgenic for the HD mutation. *Cell*.

[87] Bulone D, Masino L, Thomas DJ, San Biagio PL, Pastore A (2006). The interplay between polyQ and protein context delays aggregation by forming a reservoir of protofibrils. *PLoS One*.

[88] Nozaki K, Onodera O, Takano H, Tsuji S (2001). Amino acid sequences flanking polyglutamine stretches influence their potential for aggregate formation. *NeuroReport*.

[89] Bhattacharyya A, Thakur AK, Chellgren VM (2006). Oligoproline effects on polyglutamine conformation and aggregation. *Journal of Molecular Biology*.

[90] Masino L, Kelly G, Leonard K, Trottier Y, Pastore A (2002). Solution structure of polyglutamine tracts in GST-polyglutamine fusion proteins. *FEBS Letters*.

[91] Robertson AL, Bate MA, Buckle AM, Bottomley SP (2011). The rate of polyQ-mediated aggregation is dramatically affected by the number and location of surrounding domains. *Journal of Molecular Biology*.

[92] Robertson AL, Bottomley SP (2010). Towards the treatment of polyglutamine diseases: the modulatory role of protein context. *Current Medicinal Chemistry*.

[93] Tobelmann MD, Murphy RM (2011). Location trumps length: polyglutamine-mediated changes in folding and aggregation of a host protein. *Biophysical Journal*.

[94] Chow MKM, Ellisdon AM, Cabrita LD, Bottomley SP (2006). Purification of Polyglutamine Proteins1. *Methods in Enzymology*.

[95] Tanaka M, Morishima I, Akagi T, Hashikawa T, Nukina N (2001). Intra- and intermolecular *β*-pleated sheet formation in glutamine-repeat inserted myoglobin as a model for polyglutamine diseases. *Journal of Biological Chemistry*.

[96] Aachmann FL, Otzen DE, Larsen KL, Wimmer R (2003). Structural background of cyclodextrin-protein interactions. *Protein Engineering*.

[97] Irie T, Uekama K (1999). Cyclodextrins in peptide and protein delivery. *Advanced Drug Delivery Reviews*.

[98] Szejtli J (1998). Introduction and general overview of cyclodextrin chemistry. *Chemical Reviews*.

